# Application of BP Neural Networks in Garment Pattern Design System

**DOI:** 10.1155/2022/8766137

**Published:** 2022-05-10

**Authors:** Shuo Ma, Xiaoyu Yan

**Affiliations:** ^1^College of Fine Arts and Design, Hebei Institute of Communications, Shijiazhuang 050000, China; ^2^Faculty of Art & Design, Universiti Teknologi MARA, Shah Alam 40450, Malaysia

## Abstract

With the intensification of global market competition and the continuous development of the information technology, competition in the apparel market has become increasingly fierce. The key to whether China's garment industry can maintain its advantage in the international market competition in the future lies in whether it can promote and realize the informatization of the garment industry or not. After all, under the context of increasingly developed information technologies and growing competition in the garment market, mass customization of garments has become a future trend in the garment industry. As custom-made clothing is more in line with consumers' individual needs in terms of style, fabric, and size, the focus of development for clothing companies is increasingly on the grasp of the fit of clothing. However, with China's large population and the wide variety of body types, traditional hand-made garments are time-consuming and cannot meet the differentiated needs of consumers in the modern market. The design of garment samples is an important part of the industrial production of garments and is highly dependent on the skills and experience of the operators. In other words, the level of technical expertise can determine the quality and shape of a garment product to a certain extent. As a result, in order to further improve the efficiency and quality of garment sample design and to reduce the dependence on operator skills and experience, this study proposes an intelligent garment paper sample design system based on BP neural networks. The system mainly utilizes the self-learning, self-organizing, and adaptive as well as nonlinear mapping functions of artificial neural networks to design clothing samples autonomously, thus improving the design efficiency. In the era of rapid development of information technology and artificial intelligence technology, the development of intelligent garment pattern design systems with independent intellectual property rights is of great significance in promoting the prosperity of the garment industry.

## 1. Introduction

The garment industry was one of the earliest industries to emerge in the human history. The Industrial Revolution transformed traditional hand-made garments into a mechanized method and laid the foundations for the mass production of garments [1]. In the traditional hand-made garments, although garment patterns existed, they were few in number. However, in large-scale garment production, a certain degree of standardization is required in the production of garments [2]. As a result, the production capacity of the company must be of a certain scale, which is why the pattern is so important as a key component of garment production. At the same time, today's rapid development of information technologies has led to increased competition in the market. The development of the global economy has led to an increasing focus on individuality and fit [3]. Thus, the production of garments based on clothing samples, as a production method that meets this trend, will become a key focus of the future garment industry. After all, the current development of society has entered the era of information technology. With the development of computer technology, garment customization has become a key focus of research in the garment industry [4]. In order to better meet the psychological needs of consumers in the pursuit of individuality, some clothing companies are now producing personalized items for consumers, and such forms of production and sales will continue to emerge in the future. At the same time, from the consumer's point of view, the difference in the income level and value orientation of consumers will lead to differences in consumer needs [5]. Personalization can cater to people's desire for quality and individuality. As people's demand for personalization grows, the huge potential of the garment customization market is yet to be released [6]. However, most of the traditional clothing customization in China is a small workshop operation, which has not yet been standardised and scaled up. As a result, the introduction of industry standards is imperative to the further development of China's apparel market. With the rapid development of information technology and Internet technology, personalized design and production of clothing for consumers through computer technology will become a popular form of clothing consumption in the future [7].

The garment pattern is a standardised series of templates for the industrial production of garments based on a structural design. For a garment product, there are a variety of structural patterns, which can be divided into cutting patterns and process patterns [8]. For the whole garment production enterprise, each garment product requires a set of corresponding industrial patterns. The garment industry in China is now in an era of change, and as a result of the diversification of market consumption, the styles of garments produced are changing rapidly, and the number of industrial patterns for garments has increased dramatically. From the current actual situation of China's garment industry, the production of many garment enterprises is still based on foreign trade processing-type production. In such garment enterprises, in order to maximize companies' profits, the production departments usually try to take as many orders as possible [9]. The limited production capacity of enterprises, especially the technical departments, often results in low output, which becomes a serious problem for the development of enterprises [10]. In this type of foreign trade processing company, the garments produced are relatively homogeneous and are often produced in similar styles. As a result, if the enterprise can manage the previously produced garment samples in an orderly manner, it can greatly accelerate the efficiency of garment production [11]. In fact, compared to the intelligent production of garment samples, hand-made production is inefficient and costly. As a result, in many core areas, the accuracy of hand-made production lags behind, seriously hindering the development of scale and standardization in the industry, and making it difficult for garment customization to reach the masses [12]. Therefore, it is increasingly important to explore the transformation and upgrading of the garment customization industry, combining the idea of garment sample design with computer technology to make garment customization more efficient and convenient.

With the rapid modernization of the garment industry and the emergence of a new production model of mass customization, the success of garment products requires lower prices and shorter delivery times [13]. In this context, it is necessary for garment manufacturers to make technological changes and to introduce all-round digital management in order to upgrade the industry. As an important part of the technical preparation for the production of garments, pattern design is a difficult task that combines creativity and repetition [14]. For many years, the industry has been operating on a programmed basis, with the apprenticeship of teachers and the accumulation of experience [15]. In the face of increasingly fierce competition in the domestic and international clothing market and the rapidly changing psychology of clothing consumers, traditional design concepts and management methods have failed to meet the needs of modern industrial production [16]. Therefore, with the rapid development of computers today, the organic combination of intelligent technology and garment pattern design system can greatly promote the development of China's garment industry.

As computer technology continues to develop, expert systems [17–19], machine learning [20, 21], and other artificial intelligence technologies [22, 23] have laid a good technical foundation for clothing pattern making. Some people envisage that the future of computerized pattern making is based on the computer's recognition and understanding of clothing styles, with the computer carrying out the reasoning and judgement of pattern making and the operator only responsible for judgement and correction [24]. As the reasoning and judgement ability of the computer continues to improve, the technical level of computerized pattern making will be able to reach the technical level of the operator. In the future, the operator will be both the user and the developer, while the software developer will only be the creator and maintainer of the development platform. There has been some research into the application of artificial intelligence techniques such as neural network models and expert systems to garment pattern design. Wang et al. [25] used the method of artificial neural network to research on garment pattern design and established a BP neural network model for garment pattern design, which laid the theoretical foundation for the realization of intelligence from garment design to boarding [25]. Papachristou et al. [26] analyzed and compared traditional manual pattern making and existing CAD pattern design systems as well as proposed user-friendly functions and functional collection modules for CAD pattern design systems [26]. Ho et al. [27] introduced the modelling method of artificial neural networks, described the current status of the application of this technique in comfort research, and discussed the technical construction of comfort neural networks [27]. Celcar et al. [28] discussed the key technologies for the development of an expert system for the automatic generation of garment PDS patterns from three aspects: the description of garment structures, the acquisition of expert knowledge and the establishment of a knowledge base, and the adoption of parametric design ideas [28]. Also, they introduced in detail the implementation methods of intelligent pattern generation, such as the construction of virtual patterns and the establishment of mathematical models of patterns, using specific patterns as examples.

In short, artificial neural networks can be used to learn from the design experience of garment designers and producers. In order to change the inefficient productivity of attendants, apparel CAD needs to introduce artificial intelligence technologies, including neural networks, in order to move towards a high level of intelligence. As neural networks support a variety of intelligent technologies including self-learning and self-organization, the physical relationship between the body parameter data and the graphic key point data of the corresponding board type can be reflected in the mathematical relationship between the network input and the network output of the neural network in a garment marking system. The learned and trained network model can then be used to replace the original parametric board-making system for structural optimization and to accumulate design experience, thereby improving efficiency and avoiding interdependence between graphic data. Furthermore, this new mode can increase the intelligence of the garment pattern design system. By providing intelligent support for designers in the apparel pattern module, it enables a variety of intelligent features such as self-learning, self-correcting, associative memory, pattern recognition, and automatic knowledge acquisition. With the help of these features, the requirements for human knowledge and experience in paper pattern design can be reduced, complicating the process and lowering the employment costs of enterprises. This will undoubtedly change traditional design and greatly improve its efficiency. In addition to this, the efficiency and quality of paper prototyping work can be improved, freeing up large numbers of design technicians from repetitive work and enabling the standardization and optimization of product design.

In order to achieve rapid computer-aided garment pattern making, the efficiency and accuracy of pattern making are improved. In this study, a BP neural network algorithm is applied to capture and represent different types of clothing pattern designs and to build a knowledge base model of clothing patterns. To be specific, the knowledge will be collated to provide a comprehensive representation of the richly varied and empirical pattern design knowledge and to discover the regular knowledge in the database. After that, the knowledge can be extracted using data mining methods to achieve automatic knowledge acquisition. In particular, the list of relationships is proposed for the fuzzy knowledge in garment pattern design. Also, through the comprehensive use of multiple models, a knowledge base suitable for design requirements and a reasoning mechanism for pattern design should be established on the basis of a comprehensive analysis of the laws of garment pattern generation. This will improve the accuracy and efficiency of the garment pattern design system, thus enhancing the core competitiveness of enterprises in the garment industry.

## 2. Intelligent Garment Pattern Generation Method

For many small and medium-sized garment companies, although they may have a garment CAD system, they lack experienced pattern makers. Therefore, when the structure of the garment changes, it is important to design the appropriate pattern, and the experience of the pattern maker is particularly essential. If there is an intelligent garment pattern design system that can generate patterns directly according to the user's individual requirements, then the productivity and efficiency can be greatly increased. Although some large garment companies do not have a shortage of experienced pattern makers, some of the core skills are in the hands of these pattern makers. As a result, if they choose to leave, it can be a major problem for the company. In addition, with the existing apparel CAD system, even experienced pattern makers need to spend a lot of time designing garment patterns, which will greatly reduce the productivity and efficiency. Therefore, the creation of an intelligent garment pattern design system with automatic design and independent learning can effectively improve the productivity and efficiency of the garment industry, which is of great importance for garment companies. Some of the existing methods of automatic pattern generation are mainly geared towards garment personalization. However, in the process of automatic garment pattern structure generation, the main use of computer graphics technology is to simulate the existing garment style pattern drawing rules and methods.

### 2.1. Framework of Intelligent Garment Pattern Generation Method

Based on the above problems, this study proposes an intelligent garment pattern generation method. This approach is mainly oriented towards the conventional production methods of garment enterprises and enables the automatic generation of garment patterns. What is more, this method has an autonomous learning capability. The specific framework of the method is shown in Figure 1.

For a given garment, the pattern of a regular garment style is relatively fixed. As a result, it is relatively simple to implement automatic garment pattern generation. However, when the style changes, the corresponding garment structure also changes accordingly. If the pattern can be found, then the pattern can be generated more easily. The intelligent garment pattern generation method proposed in this study is designed to solve the problem of pattern generation after a change in the style. To be specific, for a particular garment, some parts of the pattern change can be directly derived from existing theories. Therefore, this approach is important in the process of updating garment structures.

The fact that a system has an independent learning function is an important indication of the system's intelligent nature. An important aspect of the CAD system's inability to replace the pattern maker's work is that the CAD system cannot learn the pattern maker's experience on its own. Therefore, it is important to quantify the experience of the pattern maker in an effective way. For a specific type of garment, it is first necessary to identify the parts that need to be empirically drawn, then to find the appropriate quantification method, and finally to build a self-learning proofing method using neural networks in artificial intelligence. In this case, the learning model is built to gain the experience of the pattern maker, and the corresponding garment pattern can be generated directly.

### 2.2. Design of Garment Pattern Database

The design and development of the garment pattern database are the basis and core part of the intelligent garment pattern design system, which is related to the functionality of the whole system. As a result, the design of the garment pattern database has to be based on the functions planned for the whole system to define the various function-related fields. Only by completing the design of the database according to the functional needs can the correct debugging of the relevant functions through programming be ensured later on. The intelligent garment pattern design system mainly relies on visual basic programming for its functionality, while the data are stored using a database created by Access. The database is actually used in the system and the functions for its operation are shown in Figure 2.

The functions of the intelligent garment pattern design system are closely related to the database operations. When a user adds a garment pattern, it is actually the process of adding a new record to the garment pattern database. Each time a pattern is added, a new record is added to the database. When a user retrieves a garment pattern, it is a sequential search of the data table. Deleting a pattern during database maintenance is the process of deleting a record from the database. As a result, the data transfer relationship in the implementation of the relevant functions is shown in Figure 3.

### 2.3. Principle of Intelligent Garment Pattern Generation Method

In the intelligent garment pattern design system, the knowledge, experience, and methods are summarized for each step of the garment pattern design process. A series of modules and prototypes are then used to encapsulate the garment attributes and design methods, resulting in a standardised template. By setting template constraints and introducing artificial intelligence algorithms to solve them, rapid design of garment styles can be achieved.

Suits are one of the closest types of clothing to fast consumption, with the rate of renewal and change gradually increasing. In addition to this, as the workplace and business interactions expand, the overall demand for suits is expanding and therefore the consumption base is growing. At the same time, the production pressure on clothing companies will increase. As a result, if the technology of automatic generation of suit patterns can be implemented, the efficiency and profitability of the company will be greatly improved. In this study, the design of the suit pattern is taken as an example, and the template is used to expand the suit design automatically and quickly into a structural pattern, as shown in Figure 4.

At present, the intelligent garment pattern design system still uses parametric predefinition and interactive user input to create the pattern for the fit of the suit. The lack of reasonable model construction for specific areas can lead to deformation, which can make the regular pattern differ significantly from the traditional paper pattern knowledge. This can lead to problems such as paper patterns that do not actually fit. This calls for the knowledge of the use of patterns in intelligent design to be sorted out and represented.

### 2.4. Generation of Rule Base

The process of expressing knowledge is the process of transforming knowledge and establishing constraints. This means that expert knowledge can be transformed into parametric design rules, which can then be used as a basis for building a rule base. In the area of computing, the application of knowledge is essentially the solution of a constraint, and the collection of all the methodological tools required to solve it forms a method library. The application of knowledge does not need to represent all cases, but only a collection of important features that share the same situation. In this research, the design of the garment pattern knowledge base for the suit can be broken down into different knowledge modules. Each knowledge module can be broken down into a number of submodules. For each submodule, there are a number of submodules. For each of these modules, a specific prototype processing method is used to represent the structural modelling characteristics of the module. The rules for each module are then stored together, completing the process of constructing a rule base for suit pattern design, as shown in Figure 5. As a result, when the designer is describing a garment style, the computer can find the rules for each module to help the designer conduct a rational and efficient design.

The generation and progression of rules in the system are reasoned in the form of a chain table of correspondence between conditions and conclusions, the structure of which is shown in Figure 6.

## 3. BP Neural Network in Garment Pattern Design System

A BP neural network consists of an input layer, an output layer, and an implicit layer. It belongs to a multilayer mapping network, which is based on the principle of minimum mean squared error learning for functions such as pattern recognition and adaptive control. As such, it is a learning algorithm for multilayer networks. The process of learning consists of two processes: forward propagation of the signal and inverse propagation of the error. When forward propagation is performed, the input samples are fed from the input layer, processed layer by layer in the implicit layer, and then passed to the output layer. If the actual output of the output layer does not match the desired output, then the process moves to the inverse propagation of the error. The inverse propagation of the error is the back propagation of the output error in some form through the implicit layer to the input layer, thus obtaining the error signal for each layer. This forward propagation of the signal and the backward propagation of the error are a continuous process of adjustment of the weights of the layers. The learning and training process of the neural network is therefore a continuous adjustment of the weights. This process continues until the network output error is reduced to an acceptable level.  Figure 7 shows the structure of a classical three-layer BP neural network. The application of BP neural networks in garment pattern making is based on the iterative calculation of the accuracy of the garment pattern by using BP neural networks in conjunction with the dimensions of the human body.

### 3.1. Learning Mechanism of BP Neural Network

In the garment pattern design system proposed in this research, the learning and training mechanism mainly includes the following steps (see Figure 8). Firstly, it is necessary to determine the number of layers of the BP neural network, the number of nodes in each layer, and the excitation function. Then, the weighting matrix and threshold values for each layer, the learning rate, error limits, and the maximum number of iterations will be initialized. After that, the input and target variables will be normalized and the resulting normalized data will be fed into the neural network for learning and training. Finally, the output values of the nodes in the output layer are calculated separately from the excitation function of each layer, and the error values of each layer will be calculated separately.

### 3.2. Self-Learning Mode of BP Neural Network

The foundation of self-learning mode is the study of critical control points. To be specific, the system can extract the variation data of key points through the clothing sample drawn by the designer. Then, this system can get the change rules of key points through data analysis and form the recommendation rules, so as to achieve personalized customized service for customers. When the designer draws the garment sample, the system can learn some key parts. In the BP neural network-based garment pattern design system, the number of nodes in the implicit layer has a significant impact on the performance of the system. Therefore, it is worth studying and exploring how to select the right number of nodes for the hidden layer. If the number of nodes in the implicit layer is quite small, the self-learning model will have limited learning capability and will not be able to accurately reflect the structural changes in the garment design process. Similarly, if the number of nodes in the implicit layer is quite high, not only is there a problem of overfitting the data but also the design process can take too much time, thus reducing the productivity and efficiency of designing garment patterns. As a result, the basic principle is that the number of nodes should be selected as low as possible on the basis of the correct reflection of the input and output relationship, thus reducing the complexity of the neural network and increasing the productivity and efficiency of designing the garment pattern.

At present, the number of nodes in the implicit layer needs to be calculated according to empirical rules. According to equations (1)–(4), the number of nodes corresponding to the minimum network error value is selected in this study.

(1) $$\begin{array}{c} n=\sqrt{x+y}+c, \end{array}$$

where *n* refers to the number of nodes in the implicit layer, *x* is the number of nodes in the input layer, *y* refers to the number of nodes in the output layer, and *c* is a constant.

(2) $$\begin{array}{c} n=\ln\left(c^{x}\right), \end{array}$$

(3) $$\begin{array}{c} n=\sqrt{x}, \end{array}$$

(4) $$\begin{array}{c} n=\sqrt{x}\times y. \end{array}$$

According to the estimation of the empirical rule, the range of the number of nodes in the implicit layer is 5–18.

In the BP neural networks, the transfer function in the implicit layer usually selects Sigmoid activation function. This function is smooth and differentiable. Compared with the linear function, it is more accurate, so it has better fault tolerance for neural network. The graph of this function is shown in Figure 9.

In order to solve the overfitting problems encountered in the application process and improve the training efficiency of neural network, it is necessary to normalize the input garment sample data. The range of data can be controlled between 0 and 1 through normalization, as shown in the following equation:

(5) $$\begin{array}{c} \hat{v_{i}}=\frac{v_{i}-v_{\min}}{v_{\max}-v_{\min}}, \end{array}$$

where $\hat{v_{i}}$ is the garment pattern value after normalization, *v*_*i*_ is the garment pattern value before normalization, *v*_min_ is the minimum value in the data set, and *v*_max_ is the maximum value in the data set.

## 4. Conclusion

With the rapid development of Internet technology and information technology and the development needs of modern garment enterprises, automatic generation mode of garment pattern is not only the trend of the future but also the focus of research in the industry. Although there are much research focusing on automatic garment pattern design mode, their emphases and effects are different, and the real automatic production has not been realized. The research object of this paper is garment pattern design; the focus of the research is based on BP neural network research and development of clothing pattern design system, in order to improve the efficiency of clothing enterprises design and production. With the popularization and popularization of garment CAD technology, the design of garment pattern by using advanced computer technology has become the first choice of many designers and enterprises, and it is also the core requirement of the modernization of garment industry. However, people gradually feel that the adaptability between technology and operator is highlighted, so the automatic design mode has become the focus of research. In this context, this research mainly proposes an empirical quantification method, with the combination of the quantification method and BP neural network construction to build a self-learning model of garment pattern design. This model can be used to learn the sample plate master plate making experience and used in the system of automatic plate energy. At the same time, the model can be used in the process of continuous learning and training, so as to improve the design efficiency in the update.

However, since this paper is the first time to study the experience and self-learning methods of garment pattern design system, there are still some deficiencies, which need to be further studied. To be specific, in this paper, the research on the rules of conventional garment pattern design is completed according to the existing theoretical knowledge of clothing, which can be different from that in the real world of the enterprise. Therefore, it is necessary to complete the research on the rules through the cooperation with the enterprise in the future.

## Figures and Tables

**Figure 1:** Framework of the intelligent garment pattern generation method.

**Figure 2:** Garment pattern database.

**Figure 3:** Data transfer relationship in implementation of relevant functions.

**Figure 4:** Process of intelligent garment pattern design system.

**Figure 5:** Generation of rule base.

**Figure 6:** Generation of rule base.

**Figure 7:** Structure of three-layer BP neural network.

**Figure 8:** Learning process of BP neural network.

**Figure 9:** Sigmoid activation function.

## Data Availability

The labeled data set used to support the findings of this study is available from the corresponding author upon request.
